The article "Comprehensive Analysis of Novel Genes and Pathways Associated with Osteogenic Differentiation of Adipose Stem Cells" was published in 2022. Journal: Dis Markers.

# Comprehensive Analysis of Novel Genes and Pathways Associated with Osteogenic Differentiation of Adipose Stem Cells

**DOI:** 10.1155/2022/4870981

**Published:** 2022-09-12

**Authors:** Qiuni Gao, Xiaorong Ma, Zuoliang Qi

**Affiliations:** ^1^Department of Plastic and Cosmetic Surgery, Tongji Hospital, School of Medicine, Tongji University, Shanghai 200065, China; ^2^Department of Plastic and Reconstructive Surgery, Xinhua Hospital, Kongjiang Road 1665, Shanghai 200092, China; ^3^Department of Plastic and Reconstructive Surgery, Plastic Surgery Hospital, Chinese Academy of Medical Sciences and Peking Union Medical College, No. 33 Badachu Road, Shijingshan District, Beijing 100144, China

## Abstract

**Background:**

Adipose-derived stem cells (ADSCs) are an important alternative source of mesenchymal stem cells (MSCs) and show great promise in tissue engineering and regenerative medicine applications. However, identifying the novel genes and pathways and finding the underlying mechanisms regulating ADSCs osteogenic differentiation remain urgent.

**Methods:**

We downloaded the gene expression profiles of GSE63754 and GSE37329 from the Gene Expression Omnibus (GEO) Database. We derived differentially expressed genes (DEGs) before and after ADSC osteogenic differentiation, followed by Gene Ontology (GO) functional and KEGG pathway analysis and protein-protein interaction (PPI) network analysis. 211 differentially expressed genes (142 upregulated genes and 69 downregulated genes) were aberrantly expressed. GO analysis revealed that these DEGs were associated with extracellular matrix organization, protein extracellular matrix, and semaphorin receptor binding.

**Conclusions:**

Our study provides novel genes and pathways that play important roles in regulating ADSC osteogenic differentiation, which may have potential therapeutic targets for clinic.

## 1. Introduction

Millions of patients around the world suffer from bone defects caused by tumors, infections, and trauma, and their repair and treatment are a major problem [1]. Over 10 million bone transplants are performed worldwide each year, and the number is still growing at a rate of 10% annually [2]. Presently, autologous bone transplantation and allogeneic bone transplantation are the two main surgical options for treating bone defects and nonunion [3, 4]. Autologous bone transplants are a common treatment for bone defects, but their use is limited due to their limited source, poor plasticity, and damaging to the donor site [5]. Allogeneic bone transplantation results in a significantly higher rate of postoperative complications, which has exceeded 30%, and includes fractures, insufficiency, and infections [6, 7].

The article "Comprehensive Analysis of Novel Genes and Pathways Associated with Osteogenic Differentiation of Adipose Stem Cells" was published in 2022. Journal: Dis Markers.

By creating replacements for natural bone grafts, bone tissue engineering aims to address the shortcomings [8]. As well as having the ability to form on demand, it should also easy to be prepared. Several advances have been made recently, including the development of human ADSCs that can perform paracrine functions as well as multilineage differentiation [9–11]. As a result of their properties, ADSCSs are especially useful in bone tissue engineering. Transplanting human ADSCs as a prospective treatment has recently received some attention [12, 13]. The treatment of bone trauma with autologous cells is therefore relatively promising. Transcriptional, posttranscriptional, and epigenetic factors regulate osteogenic differentiation of ADSCs [14]. A high-efficiency osteoinductive factor is also required as part of repairing bone tissue [15]. Wnt, PI3K/Akt, and MAPK signaling pathways were associated with osteogenic differentiation of ADSCs [16]. So, we have focused on developing osteoinductive factors that are effective. To uncover the molecular mechanisms of osteogenesis, further research is required.

ADSCs have become a hot spot in bone tissue engineering research because of their abundant sources and easy access to materials. However, the molecular biological mechanism of osteogenic differentiation of ADSCs has not been fully elucidated [17]. With the rapid development of big data and bioinformatics, as well as the application of ADSCs in the field of clinical medicine, some scholars have carried out RNA microarray and sequencing studies on the osteogenic differentiation of ADSCs to further explore the role of these RNAs in the osteogenesis of ADSCs [18, 19]. Molecular biological mechanisms during differentiation remains elusive. Molecular biology and functional genomics utilize microarray profiling to discover genes that are upregulated or downregulated, respectively [20, 21]. Therefore, in this study, bioinformatics methods were used to screen the differentially expressed genes and their involved signaling pathways during the osteogenic differentiation of ADSCs, in order to explore the molecular biological mechanism of potential key genes during the osteogenic differentiation of ADSCs. We first identified the differentially expressed genes (DEGs) from two microarray datasets selected from Gene Expression Omnibus (GEO) database. A bioinformatics approach was used to analyze the signaling pathway involving novel genes and to construct a protein–protein interaction (PPI) network. To sum up, this study found the potential key genes and the pathways involved in the osteogenic differentiation of ADSCs by mining the data related to the osteogenic differentiation of ADSCs in GEO database. These results may provide new ideas and a basis for further experimental studies to explore the genesis, development, and molecular biological mechanism of osteogenic differentiation of ADSCs in the future.

The article "Comprehensive Analysis of Novel Genes and Pathways Associated with Osteogenic Differentiation of Adipose Stem Cells" was published in 2022. Journal: Dis Markers.

## 2. Methods

### 2.1. Data Collection

Transcript profile data on osteogenic differentiation between ADSCSs and noninduced ADSCs were derived from NCBI GEO databases (http://www.ncbi.nlm.nih.gov/geo/).

GSE63754 (3 undifferentiated ADSCs and 3 osteogenic differentiated ADSCs) and GSE37329 (3 ADSCs and 2 ADSC-derived osteocytes) are the accession numbers for the collections. All of these ADSCSDs were collected from human tissues and underwent osteogenic induction.

### 2.2. Identification of Differentially Expressed Gene

R software and Bioconductor packages were applied to data mining and statistical analyses. The Limma package was subsequently used for identifying DEGs.

*P* < 0.05 and log2 fold change (log2FC) > 1 or < −1 were considered as the cutoff values for DEGs to be considered statistically significant. R software was used to produce heat maps of common significant differentially expressed genes between GSE63754 and GSE37329.

### 2.3. GO and KEGG Enrichment Analysis

GSEA was performed using GSEA 3.0 (http://www.broadinstitute.org/gsea/). Geneset with a *P* value less than 0.05 was considered to be significantly enriched. GO enrichment analysis was performed using the Gene Ontology Consortium Enrichment analysis tool (http://www.geneontology.org). To analyze the enriched biological processes (BPs), cellular components (CCs), molecular functions (MFs), and pathways of DEGs, GO analysis and KEGG pathway enrichment analysis were performed with the online tools DAVID (https://david.ncifcrf.gov/) and MetADSCsape (http://metADSCsape.org).

### 2.4. PPI Network Construction

STRING database (http://string-db.org) and Cytoscape software (Version 3.4.0) were used to identify 142 upregulated DEGs and 69 downregulated DEGs. The network was visualized using Cytoscape, a widely-used tool for exploring interactions among biomolecules, including proteins and genes.

### 2.5. Statistical Methods

These statistics were generated using the R software and were two-sided. *P* values less than 0.05 were considered statistically significant.

## 3. Results

### 3.1. DEGs of GSE63754 and GSE37329

Differential gene expression analyses were visualized by volcano plots. To explore the biological classification of the DEGs overlapping in the dataset, all genes were identified in the two datasets using DAVID and MetADSCsape software. The genes are commonly regulated (*P* < 0.05 and log2 fold change (log2FC) > 1 or < −1) in GSE63754. Then, we compared the gene expression profiles between ADSCSs before and after osteogenic induction by using GSEA. Figures 1(a)–1(c) show DEGs in GSE63754. Figures 1(d)–1(f) show DEGs in GSE37329.

The article "Comprehensive Analysis of Novel Genes and Pathways Associated with Osteogenic Differentiation of Adipose Stem Cells" was published in 2022. Journal: Dis Markers.

### 3.2. GO and KEGG Pathway Enrichment Analysis

Through GO and KEGG analysis, we found that DEGs of GSE63754, extracellular matrix organization, ossification, bone mineralization, regulation of inflammatory response, and bone remodeling were mainly showed enrichment in the biological process (BP) categories. As for cellular component (CC) categories, collagen-containing extracellular matrix, high-density lipoprotein particle, plasma lipoprotein particle, plasma lipoprotein particle, and protein-lipid complex were detected; and in molecular function (MF), receptor ligand activity, extracellular matrix structural constituent, growth factor activity, Wnt-protein binding, and cytokine receptor binding. With regard to KEGG pathway, cytokine-cytokine receptor interaction, ECM-receptor interaction, PI3K-Akt signaling pathway, PPAR signaling pathway, and cholesterol metabolism were the top pathways involved in the osteogenic differentiation of ADSCs (Figures 2(a)–2(d)). Gene Ontology analyses of upregulated and downregulated DEGs are listed in Tables 1 and 2.

In GSE37329 dataset, regulation of blood pressure, chemokine production, regulation of inflammatory response, regulation of chemokine production, and regulation of fat cell differentiation were detected in BP. In CC categories, we found collagen-containing extracellular matrix, synaptic membrane, presynapse, exocytic vesicle, and transport vesicle were mainly shown. As for MF, glycosaminoglycan binding, G protein-coupled peptide receptor activity, peptide receptor activity, Wnt-protein binding, and extracellular matrix structural constituent were figured out. The results of KEGG pathway demonstrated that drug metabolism-cytochrome P450, tyrosine metabolism, neuroactive ligand-receptor interaction, and vascular smooth muscle contraction were important in the osteogenic differentiation of ADSCs (Figures 2(e)–2(h)).

### 3.3. Overlapping DEGs of Datasets

The commonly and differentially expressed genes in GSE63754 and GSE37329 during osteogenic differentiation of ADSCs were identified (*P* < 0.05 and log2 fold change (log2FC) > 1 or < −1). To investigate the biological classification of the 142-overlapping upregulated DEGs and 69-overlapping downregulated DEGs, DAVID and MetADSCsape software packages were used to identify genes in the two datasets. In 142 upregulated overlapping DEGs, we found that positive regulation of secretion and positive regulation and fatty acid degradation were in the center of GO network. In 69-overlapping downregulated DEGs, striated muscle tissue development and muscle tissue development were significantly different (Figures 3(a)–3(d)).

The article "Comprehensive Analysis of Novel Genes and Pathways Associated with Osteogenic Differentiation of Adipose Stem Cells" was published in 2022. Journal: Dis Markers.

### 3.4. Key Candidate Gene Identification with DEG PPI Network

Based on the STRING online database and Cytoscape software, DEG protein–protein interaction (PPI) network complex was constructed. We collected 142-overlapping upregulated DEGs and 69-overlapping downregulated DEGs to create the PPI network. The central node genes might potentially play an important role in regulating ADSC osteogenic differentiation (Figure 4).

## 4. Discussion

In the field of tissue engineering, the use of biocompatible scaffolds has increased in recent years [22]. The ability to self-renew, the proliferation potential, and the multipotency of ADSCs make them attractive for regenerative medicine applications [23, 24]. Since ADSCs are readily available and easy to obtain in large quantities, they have become promising seed cells for bone tissue engineering [25]. In order for ADSC-based therapies to be successful in vivo, they must be paired with a substance that facilitates their osteogenic differentiation in vivo [26]. Thus, it is critical that we understand the molecular mechanisms that underlie osteogenic differentiation in ADSCSs.

We firstly analyses GSE63754 (3 undifferentiated ADSCs and 3 osteogenic differentiated ADSCs) and GSE37329 (3 ADSCs and 2 ADSC-derived osteocytes). Because of this study, we found 211 significant DEGs common to both microarrays (142 upregulated and 69 downregulated). The most enrichment is extracellular matrix organization in the BP category. The extracellular matrix is an active factor in cellular differentiation, and modifying its composition can greatly influence osteogenic differentiation of mesenchymal stem cells (Hwang et al., 2015). Other BP, such as ossification, bone mineralization, regulation of inflammatory response, and bone remodeling, were also showed enrichment. ADSCSs undergo osteogenic differentiation, thus, a regulation of genes negatively related to cell proliferation is observed.

In CC categories, collagen-containing extracellular matrix, high-density lipoprotein particle, plasma lipoprotein particle, plasma lipoprotein particle, and protein-lipid complex showed the highest enrichment score. It is interesting to note that two of the top eight CCs that are highly associated with ADSCS osteogenic differentiation are either located in the extracellular space or are located in the cell membrane, indicating that cell-to-cell signaling plays a crucial role in osteogenic differentiation. In MF categories, except chemorepellent activity, enhancer sequence-specific DNA binding, and semaphorin receptor binding, Wnt-protein binding and Wnt-activated receptor activity are most important factors. ADSCs differentiate into osteoblasts through Wnt proteins, and bone formation occurs via these proteins. It is possible that disrupting Wnt signaling pathway might significantly affect bone regeneration and remodeling [27–29]. ADSCs differ in their osteogenic differentiation in response to a variety of signaling pathways, including ERK1/2, Wnt, PI3K/Akt, and BMP-Smad. These proteins enable ADSCs to differentiate into osteoblasts and lead to bone formation. In KEGG pathway, the top significantly changed pathways of upregulated genes are related to drug metabolism-cytochrome P450, tyrosine metabolism, fatty acid degradation, cholesterol metabolism, retinol metabolism, and PPAR signaling pathway. ADSCSs that differentiate into osteoblasts have downregulated genes influenced by the adipogenesis pathway.

The article "Comprehensive Analysis of Novel Genes and Pathways Associated with Osteogenic Differentiation of Adipose Stem Cells" was published in 2022. Journal: Dis Markers.

ADSCs were targeted by several pathways which affected osteogenic differentiation and, as a result, affected bone formation. In our study, we constructed a PPI network which is composed of the associated genes. PODXL is a negatively charged sialic acid glycoprotein, belonging to the type I transmembrane glycoprotein, which has been reported to be associated with poor prognosis in oral squamous cell carcinoma, colon cancer, glioblastoma, and breast cancer and has an impact on cell adhesion and migration. It has a promoting effect, and PODXL is an important condition for maintaining the stability of the pod cytoskeleton [30]. SEMA3D is a member of the class III semaphorin family and is a marker of osteoarthritis. Class III semaphorins are involved in normal bone homeostasis and bone pathology and have a complex relationship between osteoblasts and osteoclasts which has the potential to treat bone disease [31]. The ADGRG6 single nucleotide polymorphism is associated with human height, and its deletion in osteoblasts may delay osteoblast differentiation and bone formation, resulting in shortened body length and reduced bone mass in mice [32–34]. CADM3 is an immunoglobulin adhesion molecule belonging to the Nectin molecule-like family of proteins [35]. The constitutive expression level of RERG in calvaria was 1000-fold higher than in femoral osteoblasts; during osteogenic induction, RERG expression was downregulated in calvarial osteoblasts and upregulated in femoral osteoblasts [20]. The osteocytes of the skull are fundamentally different from those of the femur and respond differently to a range of stimuli. These site-specific differences may have important implications in developing strategies to address metabolic bone disease [36]. APCDD1 is an inhibitor of Wnt signaling pathway, which can promote the adipogenic differentiation and lipid anabolism of bone marrow stromal cells [37]. NRCAM may modulate geometric parameters of the femoral neck and contribute to an improved understanding of osteoporosis and pathophysiological mechanisms [38, 39]. The target genes supported by these literatures are related to bone homeostasis, osteogenic differentiation, bone diseases, and metabolism, which supports the feasibility of this study to explore the underlying molecular mechanisms during the osteogenic differentiation of adipose-derived stem cells [40].

The article "Comprehensive Analysis of Novel Genes and Pathways Associated with Osteogenic Differentiation of Adipose Stem Cells" was published in 2022. Journal: Dis Markers.

The drawback of our study is the lack of functional cellular and animal experiments for validation to explore the occurrence, development, and molecular biology of osteogenic differentiation of ADSCs. In conclusion, based on two transcript profile data on osteogenic differentiation between ADSCs and noninduced ADSC datasets and comprehensive analysis, we have identified several genes and pathways that could be crucial to osteogenic differentiation of ADSCs. Understanding of how ADSCs differentiate into osteoblasts could be improved significantly by our new findings. Moreover, manipulation of these genes and pathways may lead to bone regeneration and tissue engineering.

## Figures and Tables

**Figure 1:** DEGs of GSE63754 and GSE37329. (a–d) Volcano plot: the volcano plot was constructed using the fold change values and *P*-adjust. Red dots indicate upregulated genes; blue dots indicate downregulated genes. (c–f) Gene set enrichment analysis (GSEA) of two significantly enriched classes of genes: ADSCs and noninduced ADSC datasets.

**Figure 2:** GO and KEGG pathway enrichment analysis. (a–h) Gene Ontology (GO) analysis and enriched KEGG signaling pathways were selected to demonstrate the primary biological actions of major potential genes. Colors represent the significance of differential enrichment, the size of the circles represents the number of genes, the larger the circle, the greater the number of genes. In the enrichment result, *P* < 0.05 or FDR < 0.05 is considered to be a meaningful pathway (enrichment score with −log10 (*P*) of more than 1.3). BP: biological process; CC: cellular component; MF: molecular function.

**Figure 3:** Overlapping DEGs of datasets. (a–d) Gene Ontology (GO) analysis and enriched KEGG signaling pathways were selected to demonstrate the primary biological actions of major potential genes. Colors represent the significance of differential enrichment, the size of the circles represents the number of genes, the larger the circle, the greater the number of genes. In the enrichment result, *P* < 0.05 or FDR < 0.05 is considered to be a meaningful pathway (enrichment score with −log10 (*P*) of more than 1.3). BP: biological process; CC: cellular component; MF: molecular function.

The article "Comprehensive Analysis of Novel Genes and Pathways Associated with Osteogenic Differentiation of Adipose Stem Cells" was published in 2022. Journal: Dis Markers.

**Figure 4:** Key candidate gene identification with DEG PPI network. PPI network of the common significant differentially expressed genes was constructed. A total of 142-overlapping upregulated DEGs and 69-overlapping downregulated DEGs were identified by Cytoscape. PPI: protein–protein interaction.

**Table 1:** Gene Ontology analyses of upregulated DEGs.

Ontology	ID	Description	GeneRatio	BgRatio	*P* value	*P*.adjust	*Q* value
BP	GO: 1903532	Positive regulation of secretion by cell	13/130	399/18670	4.36e-06	0.009	0.008
BP	GO: 0051047	Positive regulation of secretion	13/130	428/18670	9.27e-06	0.009	0.008
BP	GO: 0002532	Production of molecular mediator involved in inflammatory response	6/130	72/18670	1.09e-05	0.009	0.008
BP	GO: 0070542	Response to fatty acid	6/130	86/18670	3.03e-05	0.014	0.012
BP	GO: 0050727	Regulation of inflammatory response	13/130	485/18670	3.44e-05	0.014	0.012
CC	GO: 0034358	Plasma lipoprotein particle	4/134	37/19717	1.13e-04	0.012	0.011
CC	GO: 1990777	Lipoprotein particle	4/134	37/19717	1.13e-04	0.012	0.011
CC	GO: 0032994	Protein-lipid complex	4/134	39/19717	1.39e-04	0.012	0.011
CC	GO: 0099061	Integral component of postsynaptic density membrane	4/134	50/19717	3.69e-04	0.017	0.015
CC	GO: 0099146	Intrinsic component of postsynaptic density membrane	4/134	53/19717	4.61e-04	0.017	0.015
MF	GO: 0016709	Oxidoreductase activity	4/130	39/17697	1.87e-04	0.065	0.058
MF	GO: 0004745	Retinol dehydrogenase activity	3/130	20/17697	4.03e-04	0.070	0.063
MF	GO: 0004497	Monooxygenase activity	5/130	99/17697	8.16e-04	0.094	0.084
KEGG	hsa00982	Drug metabolism-cytochrome P450	8/66	71/8076	9.12e-08	1.48e-05	1.40e-05
KEGG	hsa00350	Tyrosine metabolism	5/66	36/8076	9.69e-06	7.85e-04	7.45e-04
KEGG	hsa00071	Fatty acid degradation	4/66	44/8076	4.32e-04	0.023	0.022
KEGG	hsa04979	Cholesterol metabolism	4/66	50/8076	7.07e-04	0.029	0.027
KEGG	hsa00830	Retinol metabolism	4/66	68/8076	0.002	0.073	0.069

**Table 2:** Gene Ontology analyses of downregulated DEGs.

Ontology	ID	Description	GeneRatio	BgRatio	*P* value	*P*.adjust	*Q* value
BP	GO: 0010721	Negative regulation of cell development	12/66	344/18670	2.55e-09	5.10e-06	3.85e-06
BP	GO: 0060537	Muscle tissue development	12/66	408/18670	1.71e-08	1.71e-05	1.29e-05
BP	GO: 0014706	Striated muscle tissue development	11/66	390/18670	1.10e-07	7.34e-05	5.54e-05
BP	GO: 0050768	Negative regulation of neurogenesis	9/66	295/18670	9.14e-07	4.57e-04	3.45e-04
BP	GO: 0051961	Negative regulation of nervous system development	9/66	315/18670	1.57e-06	6.29e-04	4.75e-04
CC	GO: 0005913	Cell-cell adherens junction	4/66	117/19717	6.39e-04	0.026	0.024
CC	GO: 0045121	Membrane raft	6/66	315/19717	6.44e-04	0.026	0.024
CC	GO: 0098857	Membrane microdomain	6/66	316/19717	6.55e-04	0.026	0.024
CC	GO: 0098589	Membrane region	6/66	328/19717	7.95e-04	0.026	0.024
CC	GO: 0016342	Catenin complex	2/66	29/19717	0.004	0.092	0.084
MF	GO: 0045499	Chemorepellent activity	4/63	27/17697	2.41e-06	5.22e-04	4.61e-04
MF	GO: 0001158	Enhancer sequence-specific DNA binding	5/63	119/17697	6.50e-05	0.005	0.005
MF	GO: 0030215	Semaphorin receptor binding	3/63	23/17697	7.24e-05	0.005	0.005
MF	GO: 0035326	Enhancer binding	5/63	133/17697	1.10e-04	0.006	0.005
MF	GO: 0005539	Glycosaminoglycan binding	6/63	229/17697	1.61e-04	0.007	0.006
KEGG	hsa04550	Signaling pathways regulating pluripotency of stem cells	5/40	143/8076	6.48e-04	0.064	0.061
KEGG	hsa04350	TGF-beta signaling pathway	4/40	94/8076	0.001	0.064	0.061

The article "Comprehensive Analysis of Novel Genes and Pathways Associated with Osteogenic Differentiation of Adipose Stem Cells" was published in 2022. Journal: Dis Markers.

## Data Availability

All the data in this manuscript can be acquired by request.
